# Prediction of Cancer-Specific Survival of Brainstem Glioma in Children Based on Risk Stratification Model

This article has been retracted.

**DOI:** 10.1155/2022/3436631

**Published:** 2022-07-20

**Authors:** Kai Sun, Mingwei Xu, Xiaowei Fei, Hao Wang, Lunshan Xu, Ruxiang Xu, Minhui Xu

**Affiliations:** ^1^Department of Neurosurgery, Daping Hospital, Army Medical University, Chongqing 400042, China; ^2^Department of Neurosurgery, Sichuan Academy of Medical Sciences and Sichuan Provincial People's Hospital, School of Medicine, University of Electronic Science and Technology of China, Chengdu, Sichuan 610072, China; ^3^Department of Neurosurgery, The First Affiliated Hospital of The Fourth Military Medical University, Xi'an, Shaanxi, 710032, China

## Abstract

**Objective:**

To develop and authenticate a risk stratification framework and nomogram for ascertaining cancer-specific survival (CSS) among the pediatric brainstem gliomas.

**Methods:**

For patients less than 12 years, according to Surveillance, Epidemiology, and End Results (SEER), information from 1998 to 2016 is found in their databases. The survival outcomes, treatments, and demographic clinicopathologic conditions are scrutinized per the database validation, and training cohorts are divided and validated using multivariate Cox regression analysis. A nomogram was designed, and predominantly, the risk stratification conceptualization engaged selected tenets according to the multivariate analysis. The model's authenticity was substantiated through C-index measure and calibration curves.

**Results:**

There are 806 pediatric concerns of histologically concluded brainstem glioma in the research. According to multivariate analysis, age, grade, radiotherapy, and race (with *P* value < 0.05) depicted independent prognostic variations of the pediatric gliomas. The nomogram's C-index was approximately 0.75 and an accompanied predictive capability for CSS.

**Conclusion:**

The nomogram constructed in this glioma's context is the primary predictor of using risk stratification. A combination of nomograms with the risk stratification mechanism assists clinicians in monitoring high-risk individuals and engage targeted accessory treatment.

## 1. Introduction

Gliomas are common intracranial primary malignancies, accounting for 35.26% to 60.96% of all central nervous system tumors, with a high degree of malignancy, and the fatality rate ranks 2nd and 3rd in malignant tumors in people aged ≤34 years and 35 to 54 years old, respectively [1]. Gliomas are a type of neuroepithelial tumor that arises from the central nervous system's glia or supporting cells (astrocytes, oligodendrocytes, and ependymocytes) [2–4]. Gliomas account for almost a quarter of all recurrent brain and CNS tumors and range in histopathology and conduct from simple ependymal tumors to the worst aggressive and deadly grade IV glioblastoma multiforme [5, 6]. Among them, grades I~II and III-IV are low-grade glioma (LGG) and high-grade glioma (HGG), respectively, and there are obvious differences in the treatment plan and prognosis of patients at different levels, so early accurate diagnosis and grading are extremely important for glioma treatment [7]. The detailed cause is not yet clear, and previous studies believe it may be closely related to factors such as genetics, infection, and environmental pollution. Brainstem gliomas comprise limited localized brainstem gliomas and high-grade distributed inherent pontine gliomas (DIPGs), which are a heterogeneous category of neoplasms that mostly affect children [8–12]. The remaining low-grade gliomas are found in the midbrain, dorsal medulla, or cervical-medullary junction, even though 80 percent of gliomas begin as DIPGs in the pons. These neoplasms' sites, as indicated, provide therapeutic obstacles and may harm treatment.

Surgical resection is the main treatment at this stage, and postoperative adjuvant chemoradiation also positively affects prolonging survival time. The standard therapeutic choices for gliomas are radiotherapy, chemotherapy, and combination treatment modalities [11, 13]. Previous research has shown that chemotherapy fails to treat DIPGs due to a lack of tumor penetration [6, 14, 15]. The finding of the K27M mutation (mutation in both histones H3.1 and H3.3) and the unraveling of the genetic landscape of DIPGs have recently offered further knowledge on the etiology of gliomas and the identification of potential targeted therapies [6, 16, 17].

Despite the abundance of data on cancer staging, survival prediction, and treatment methods, little is known about cancer-specific survival (CSS) factors in children with brain stem gliomas. Surveillance, Epidemiology, and End Results (SEER) is a repository of survival statistics from community-based cancer registries covering about 28% of the US population [18–23]. This work is aimed at creating a complete, accurate, and helpful prognostic model for pediatric stem glioma cases utilizing a population-based SEER analysis to predict survival.

## 2. Material and Methods

### 2.1. Ethical Approval

This was a population study with anonymized data and was therefore exempt from ethics declaration because the research was believed not to engage human subjects.

### 2.2. Patient Selection and Study Design

The SEER-18 cohort, which included 18 cancer centers from around the United States, was used in this population analysis. This survey covered pediatric patients (ages 12 and up) with histologically diagnosed glioma identified between 1998 and 2016. Inclusion criteria are as follows: (1) complete clinical data, including clinical records and imaging tests, and (2) exclude other brain tumor cases. Exclusion criteria are as follows: (1) data from patients with missing clinical information, therapeutic details, or inadequate follow-up were excluded; (2) instances in which the brainstem was not the prime location of the lesion were also eliminated (Figure 1); and (3) patients with incomplete clinical data. The National Cancer Institute's SEER∗Stat algorithm (version 8.3.5) was used to retrieve the data. This study consists of retrospective and prospective patient profiles, tumor features, and survival results.

### 2.3. SEER-Coding and Variable Characterizations

Age at assessment, sex, and ethnicity were divided into three categories: White/Caucasian, Black/African American, and others. Histologic grade, stage, and tumor size were all factors in tumor features. Tumors were classified as large (greater than 3 cm), small (less or equal to 3 cm), or unidentified size based on the median value of the highest tumor dimensions in any study sample. The SEER database was used to get information on the treatment course, which included radiation, chemotherapy, and surgical resection other than biopsy. The diagnosis age was split into 10-year phases (1998–2008 and 2009–2016) and used as a covariate variable.

### 2.4. Statistical Designs

The chi-squared test was applied to compare continuous (rates) and categorical variables (histological grade and stage of gliomas). The survival disparity of the factors was determined using Kaplan-Meier plots. Univariate and multivariate analyses were done to identify prognostic risk factors using Cox regression. The input for multivariate analysis utilizing the Cox risk regression framework with backward exclusion was clinically significant factors that demonstrated significance (*P*0.1) in the univariate analysis. Variables that demonstrated significance (*P*0.0001) in the multivariate analysis were chosen for the nomogram. At 1, 3, and 5 years, CSS was determined. The C-index and calibration curves generated after 1000 bootstrap resampling were used to assess the nomogram's precision. Decision curve analysis is a primary benefit analysis that equivalences the accurate-positive to the weighted inaccurate-positive rates across diverse risk edges that a clinician/patient might want to accept. Based on the median value of the total nicks in the nomogram, a risk stratification model was built and comprised of patients divided into two prognostic groups. All statistical analyses were performed using R (R Foundation for Statistical Computing, Vienna, Austria) and Empower Stats (http://www.empowerstats.com, XY Solutions, Inc. Boston MA). Statistical significance was defined as a two-tailed *P* value of <0.05.

## 3. Results

### 3.1. Patient Characteristics

The participants' clinicopathological factors and demographic characteristics are sampled in Table 1. A total of 1707 participants were sampled, and 901 of the total were excluded, according to Figure 1. Ultimately, 806 pediatric issues with a histologically were situated with a diagnosis of brainstem glioma. From a range of 1 to 12 years, the median age of the participants was 6 years. The patients were composed of (74%, 596) Whites, Blacks/African Americans (17.1%, 138), and from different ethnic groups (8.9%, 72). Boys (*n* = 389, 48.3%) and girls (*n* = 417, 51.7%) showed relatively similar distributions.

The tumor size was small (≤3 cm) in 87 (10.8%), large (>3 cm) in 265 (32.9%), and unknown in 454 (56.3%) of the 806 patients. The histological grade of most tumors was unknown (*n* = 739; 91.7%). Most tumors (*n* = 720; 89.3%) were in the localized stage. Regarding treatment, radiotherapy was the utmost common treatment (*n* = 567, 70.3%), followed by chemotherapy (*n* = 360, 44.7%); only 25 (3.1%) underwent surgical resection. The median check-up duration was 11 months. Of the total, 566 (70%) patients were randomly selected and designated as the training cohort, and the remaining 240 (30%) formed the internal validation cohort (Table 1).

### 3.2. Independent Prognostic Components during Training Regiment

CSS was found to have a significant relationship with age at diagnosis, race, sex, tumor volume, histologic quality, historical stage, chemotherapy, and radiotherapy in a univariate Cox regression study. As a result, these covariates were used as input for a multivariate Cox regression analysis, which revealed that age, ethnicity, tumor magnitude, grade, and radiation were all independent predictive predictors (*P* < 0.05) (Table 2).

### 3.3. Constructing and Confirming a Nomogram

The size of the tumor, ethnicity/race, grade, radiotherapy, and age was incorporated in making a nomogram for predicting the patient's CSS, whereby *P* was less than 0.05 (see Figure 2). Every independent factor was scored on a point scale alliance. The real measure calculated as the sum of each score was weighed on the bottom scale, and the 1-, 3-, and 5-probability years for participants' CSS were estimated.

The C-index of the construct was 0.75, which demonstrated a relatively high predictive ability. Calibration plots of the nomogram (Figure 3) showed a pact between the projected CSS and actual observations. Decision curve analysis was used to determine the predictive performance for the probability of cancer-specific survival. The decision curve analysis evaluated the 1-, 3-, and 5-year CSS of children with stem glioma, which showed that all representations had a well net advantage and increased cancer-specific survival probability compared to the “treat all” approach (Figure 4).

### 3.4. Risk Stratification System

Kaplan-Meier survival analysis of age, radiotherapy, histologic grade, tumor size, and historic stage showed significant differences in survival rates (Figures 5(a)–5(e)). The total predicted score calculated from the nomogram was used in a risk stratification system to predict patient survival. Patients were grouped into those with low (total score < 130.78) and high (total score ≥ 130.78) risks. The median existence of the entire unit of patients with minimum risk and maximum risk was 24 and 7 months, respectively. The Kaplan-Meier survival curves predicted by the nomogram were significantly different (Figure 5(f)).

## 4. Discussion

For a long time, glioma has been considered to be a difficult to remove surgical and poor prognosis of intracranial tumors. Although there is current rapid development of neurosurgical techniques and radiotherapy and chemotherapy, the survival time of glioma patients has not improved significantly. Therefore, it is important to analyze the factors associated with the survival time of gliomas to guide clinical work. Though several analyses have produced nomograms for forecasting outcomes in patients with brainstem glioma, the number of observations was modest, and the prognostic parameters measured were limited [22, 24]. As a result, we created a clinical nomogram centered on the SEER database to estimate survival. The SEER registry is the most extensive individual-based database of cancer patients in the United States, including data on around 26% of all cancer patients. We used the tight scope of the study to evaluate patient data from the most recent edition of the SEER, which was initially scheduled (encompassing 18 registries from 1973 to 2015). This was necessary because the traditional staging classification, commonly used for survival prediction and clinical strategies for cancer patients, cannot accurately and consistently distinguish the difference in survival among various stages. The nomogram is a comprehensive, accurate, and useful predictive model that has been used for many types of malignancies [25]. In this study, five independent prognostic factors, age, race, tumor size, grade, and radiotherapy, identified through univariate and multivariate Cox regression analyses, were engaged in the clinical nomogram. This is consistent with the results of previous studies [26].

According to the nomogram, the tumor histology grade substantially impacted the prognosis. This discovery is similar to, but not identical to, findings from prior research on glioma survival risk factors, which found that poorly differentiated and undifferentiated histologists were strongly linked to a poor prognosis in children with brainstem glioma. Most individuals with low-grade gliomas are treated with surgery, followed by radiotherapy. However, in this trial, we discovered that radiation provided no survival benefits for young patients with brainstem gliomas. This may be related to the patient's younger age and poor tolerance to radiation therapy [27]. Chemotherapy was also ineffective in improving outcomes in cases recovered from the SEER database [22, 28–30]. Race substantially affected patient survival, with white people having higher median survival times than black persons. Whites, regardless of Hispanic status, had the highest incidence of brainstem HGG, which is similar to incidence patterns of glial tumors in general. While these differences likely reflect true predominance in these population, incidence rates may be biased towards higher reporting in non-Hispanic Whites given previous reports of their greater access to care and earlier diagnosis [31]. It was important to verify discriminatory practices using the C-index and calibration, which was examined by contrasting the compatibility between the theoretical and measured survival of patients [32–35], to confirm the nomogram and ensure that the algorithm could be deployed broadly and improve the classification accuracy. Compared to the previous staging approach, our nomogram was more effective at discriminating and predicting survival. Furthermore, according to the selection curve study, our model demonstrated a better clinical net benefit throughout all borderline probabilities [6, 36, 37]. CSS could be distinguished in children with stem glioma using the risk stratification approach performed on the two-risk population of subjects.

The nomogram is an accurate and precise prognostic approach that can help doctors identify more significant patients for personalized adjuvant treatment, especially for our dataset type [38–40]. Our research, unfortunately, had several drawbacks. First, while we used multivariable analyses to reduce confounding effects caused by variabilities, this was a retrospective study that was further hampered by the small sample size; this must be considered when considering the results [41]. Second, it is possible that the retrospective review brought selection bias into the study design [24]. Third, the SEER database is missing information on contemporary gene-array technology and molecular biomarkers such as IDH1/TERT expression [41], linked to CSS in infants with brainstem glioma. Therefore, future prospective analyses are warranted to envisage the survival of pediatric patients with gliomas.

## 5. Conclusion

The proposed study's unique nomogram for assessing the survival of hospitalized pediatric patients with patients diagnosed with brainstem glioma incorporates risk stratification for perhaps the first time. As a result, integrating the nomogram and risk classification system is a helpful tool for clinicians in locating potential patients and administering tailored antiretroviral chemotherapy.

## Figures and Tables

**Figure 1:** Patient selection of pediatric patients with brainstem gliomas within the SEER database.

**Figure 2:** Nomogram predicting 1-, 3-, and 5-year cancer-specific survival (CSS) for pediatric brainstem glioma patients.

**Figure 3:** Calibration curves predicting 1-, 3-, and 5-year cancer-specific survival (CSS) in the (a–c) training and (d–f) validation cohorts.

**Figure 4:** Decision curve analysis to determine the predictive performance for the probability of (a) 1-, (b) 3-, and (c) 5-year cancer-specific survival. The horizontal black line represents the assumption that no patient should take the necessary measures, while the gray inverse curve represents the assumption that all patients should take the necessary measures. The *y*-axis represents the net benefit, which was calculated by adding points associated with benefits and subtracting those associated with harms.

**Figure 5:** Kaplan-Meier curves of pediatric patients with brainstem gliomas in terms of (a) age, (b) radiotherapy, (c) histologic grade, (d) tumor size, (e) historic stage, and (f) risk stratification level.

**Table 1:** Patient demographics and clinicopathological characteristics of the study population.

Factors	Entire cohort (*n* = 806)		Training cohort (*n* = 566)		Validation cohort (*n* = 240)	
	*N*	%	*N*	%	*N*	%
Age at diagnosis, years						
Median	6		6		6	
Range	0–12		0–12		0–12	
Race						
White	596	74.0	426	75.3	170	70.8
Black	138	17.1	101	17.8	37	15.4
Other	72	8.9	39	6.9	33	13.8
Sex						
Male	389	48.3	278	49.1	111	46.2
Female	417	51.7	288	50.9	129	53.8
Year of diagnosis						
1998–2008	457	56.7	311	54.9	146	60.8
2009–2016	349	43.3	255	45.1	94	39.2
Tumor size, diameter, cm						
≤3	87	10.8	54	9.5	33	13.8
>3	265	32.9	197	34.8	68	28.3
Unknown	454	56.3	315	55.7	139	57.9
Histologic grade						
Well-differentiated	10	1.24	8	1.4	2	0.8
Moderately differentiated	25	3.1	17	3	8	3.3
Poorly differentiated	10	1.24	7	1.24	3	1.3
Undifferentiated	22	2.73	16	2.8	6	2.5
Unknown	739	91.7	518	91.5	221	92.1
Stage						
Localized	720	89.3	506	89.4	214	89.2
Regional	76	9.4	51	9.0	25	10.4
Distant	10	1.2	9	1.6	1	0.4
Surgery						
None	781	96.9	551	97.3	230	95.8
Yes	25	3.1	15	2.7	10	4.2
Radiotherapy						
None	239	29.6	169	29.9	70	29.2
Yes	567	70.4	397	70.1	170	70.8
Chemotherapy						
None	446	55.3	310	54.8	136	56.7
Yes	360	44.7	256	45.2	104	43.3
Median follow-up, months	11		11		11	

**Table 2:** Univariate and multivariate analyses for the training cohort.

Factors	Univariate analysis			Multivariate analysis			Score
	HR	95% CI	*P* ^∗^	HR	95% CI	*P* ^∗∗^	
Age at diagnosis, years							
≤6	1			1			16
>6	0.6	0.5–0.8	<0.001	0.8	0.6–1.0	**0.030**	0
Race							
White	1			1			5
Black	0.9	1.0–1.2	0.037	0.8	1.1–1.2	**0.035**	3
Other	1.4	0.9–2.0	0.111	0.6	0.3–2.1	0.375	0
Sex							
Male	1			1			
Female	1.3	1.0–1.5	0.028	1.1	0.9–1.3	0.586	
Year of diagnosis							
1998–2008	1						
2009–2016	0.9	0.8–1.2	0.568				
Tumor size, diameter, cm							
≤3	1			1			0
>3	4.6	2.8–7.6	<0.001	1.9	1.1–3.1	**0.013**	4
Unknown	2.8	1.7–4.5	<0.001	1.7	1.0–2.8	**0.037**	7
Histologic grade							
Well-differentiated	1			1			0
Moderately differentiated	0.7	0.2–3.0	0.669	0.8	0.2–3.1	0.722	3
Poorly differentiated	3.4	0.9–13.2	0.075	1.5	2.1–5.8	**0.021**	5
Undifferentiated	4.8	1.4–16.6	0.013	2.1	0.6–7.3	0.248	8
Unknown	2.1	0.7–6.7	0.189	1.3	0.4–4.0	0.682	10
Stage							
Localized	1			1			
Regional	1.4	1.0–1.9	0.068	1.2	0.9–1.7	0.292	
Distant	2.4	1.2–4.7	0.009	1.5	0.7–2.9	0.275	
Surgery							
None	1						
Yes	0.6	0.3–1.2	0.164				
Radiotherapy							
None	1			1			0
Yes	5.9	4.3–8.2	<0.001	4.7	3.3–6.6	**<0.001**	100
Chemotherapy							
None	1			1			
Yes	1.8	1.5–2.3	<0.001	1.0	0.8–1.3	0.779	

Bold text indicates significant variable (*P* < 0.05). Abbreviation: HR: hazard ratio.

## Data Availability

No data were used to support this study.
